RETRACTED

# Relieving the Incompatibility of Network Representation and Classification for Long-Tailed Data Distribution

**DOI:** 10.1155/2021/6702625

**Published:** 2021-12-27

**Authors:** Hao Hu, Mengya Gao, Mingsheng Wu

**Affiliations:** ^1^Postgraduate Department, China Academy of Railway Science, Beijing 100081, China; ^2^Sensetime, Beijing 100080, China; ^3^Institute of Computing Technologies, China Academy of Railway Science Corporation Limited, Beijing 100081, China

## Abstract

In the real-world scenario, data often have a long-tailed distribution and training deep neural networks on such an imbalanced dataset has become a great challenge. The main problem caused by a long-tailed data distribution is that common classes will dominate the training results and achieve a very low accuracy on the rare classes. Recent work focuses on improving the network representation ability to overcome the long-tailed problem, while it always ignores adapting the network classifier to a long-tailed case, which will cause the “incompatibility” problem of network representation and network classifier. In this paper, we use knowledge distillation to solve the long-tailed data distribution problem and fully optimize the network representation and classifier simultaneously. We propose multiexperts knowledge distillation with class-balanced sampling to jointly learn high-quality network representation and classifier. Also, a channel activation-based knowledge distillation method is also proposed to improve the performance further. State-of-the-art performance on several large-scale long-tailed classification datasets shows the superior generalization of our method.

## 1. Introduction

Commonly used datasets in the literature for CNN's training, like CIFAR [1] and ImageNet [2], are usually artificially designed and rarely suffer from the data imbalance. However, in the open real world, the distribution of data categories is often long-tailed, in which the number of training samples per class varies significantly from thousands of images to few samples. For example, in the scenarios such as railway traffic, mesothelioma diagnosis, and industrial fault detection [3, 4], we need to detect an unexpected object where the real samples for the category of unexpected object are usually hard to collect, which leads to a long-tailed data distribution. There are many works [5, 6] proposed to solve such real-world classification problems. However, they do not provide a general solution to such a long-tailed distribution problem. In this paper, we propose a general knowledge distillation-based method, which can be applied to all the long-tailed scenes.

Authors in [7, 8] also pointed out the problem that the data distribution will hardly influence the performance of deep neural network. When deep models are trained in such imbalanced scenarios, standard approaches usually fail to achieve satisfactory results, leading to a significant drop in performance. This is because that classes with more training instances, called head classes, will dominate the training procedure and the learned model tends to perform better on these classes but achieves fairly worse results for tail classes, which have very few samples [9–11]. In the literature of solving a long-tailed problem, authors in [11, 12] summarize that methods for long-tailed classification are mainly beneficial into two aspects: representation learning and classifier learning. Specifically, using some specially designed losses [13, 14] or transferring knowledge from head class [15] is helpful for tail class to learn high-quality representations and boosts model performance. Dataset resampling strategy [9, 16–19], which is to achieve a balanced data distribution, is helpful to directly influence the classifier weights and promotes the classifier learning.

RETRACTED

Although these approaches have good results eventually, they cannot optimize well representation and classifier simultaneously that some methods only focus on enhancing representation learning but taking no care of classifier learning and other methods pay attention to promoting classifier learning but will affect its representation learning ability. Authors in [11, 12] try to tackle with this problem by separating the whole training process into two stages: one for achieving good representations and the other for optimizing classifier based on the model in the first stage. However, there is no one-stage solution, which can jointly learn the two aspects well. In this paper, we define the problem as “incompatibility” between network representation learning and classifier learning, where the two aspects are hard to be optimized simultaneously, and propose a jointly learning solution.

Discovering that among different data rebalancing strategies, a class-balanced [9, 19] strategy learns a fine classifier but will affect representation learning. We propose to relieve the “incompatibility” problem by using a class-balanced strategy to achieve a good classifier and applying knowledge distillation to eliminate its weakness simultaneously. A distillation mechanism helps our CNN model to improve its representation learning ability and relieve its conflicts with classifier learning when applying class-balanced sampling.

For clarity, we define models, which have better representations for head/tail classes as experts and they will be used as teacher models in the distilling process. Specifically, we will design several teacher models that are experts for different classes (head/tail class) and then distill all expert models into one model achieving representations that performs good on both head and tail classes. Different from the aforementioned head-to-tail transfer strategy [19, 20], which takes knowledge learned from head classes as the teacher, our experts not only contain models with good representation from dominant classes but also contain those from minority classes.

RETRACTED

Furthermore, considering the representation map of a well-trained model, not all channels are highly activated when applying the input to the network. We argue that the weakly activated channels contain less information or even noise, which provide little help to the knowledge distillation process. To some extent, the useless information shared by low activation channels will affect our student to learn beneficial knowledge. As a result, we propose channel activation-based knowledge distillation to make full use of highly activated channels and discard information from the rest inactive channels.

Both multiexperts knowledge distillation and channel activation-based distillation strategy will largely boost the classification performance on the long-tailed dataset and properly solve the “incompatibility” problem, as discussed before.

Finally, to demonstrate the effectiveness of our method, we conduct exhaustive classification experiments on ImageNet-LT [10], Places-LT [10], and iNaturalist-2018 [21]. Our approach achieves outperforming results compared with existing state-of-the-art methods for long-tailed classification.

Our contributions can be summarized as follows:

- We explore the problem that in the literature of solving long-tailed data distribution problem, there exists the “incompatibility” problem between learning network representation and network classifier.
- We propose a multiexperts knowledge distillation method to solve the long-tail data problem, which can take care of representation learning and classifier learning simultaneously. Furthermore, a novel channel activation-based distillation strategy is developed for boosting the effectiveness of representation learning from the teacher model.
- We evaluate our proposed method on three large-scale long-tailed datasets and our approach consistently achieves superior performance over previous competing approaches.

## 2. Related Works

### 2.1. Long-Tailed Recognition

A long-tailed learning problem has attracted increasing attention due to the prevalence of imbalanced data distribution in real world [10, 19, 22–25]. Previous methods tackle this problem mainly from the following ways:

*Rebalancing* methods are adopted to achieve a more balanced data distribution through oversampling data for minority (tail) classes [16–18], undersampling dominant (head) classes by removing data [26, 27], and class-balanced sampling based on the number of data samples in each class [28, 29]. But sometimes resampling long-tailed dataset might lead to problems such as overfitting over rare classes or impairing generalization ability of the deep neural networks. Recently, some two-stage fine-tuning strategies were proposed to improve the effectiveness of rebalancing. Specifically, they separated the training process into two phases [11, 12]. In the first stage, the networks are trained as usual with original unbalanced data and rebalancing is applied in the second stage to fine-tune the network with few epochs and small learning rate.

RETRACTED

*Metric loss learning* aims to assign different losses for various training samples in each class. Among these methods, reweighting [9, 30] approaches allocate larger weights for tail classes to calculate training losses. Range Loss [14] enforces the distance of data from the same class to be closer and those in different classes to be far apart to improve long-tailed scenarios. Focal Loss [13] assigns lower weights for well-classified instances to deal with class imbalance. Meta-Weight-Net [31] is capable of adaptively learning an explicit weighting function directly from the unbalanced data.

*Head-to-tail class transfer* is employed to transfer knowledge learned from head classes to tail classes, which have limited samples to learn good results. The transferred knowledge, from dominant classes to minority classes, includes a transformation of regressors or classifiers [19, 20], intraclass variance [32], and deep semantic features [10], in recent works.

### 2.2. Knowledge Distillation

Knowledge distillation (KD) is first introduced in [33] and then brought back to popularity by Hinton et al. [34]. The rational behind is to use a student model (**S**) to learn from a teacher model (**T**) without sacrificing much accuracy. Existing methods have designed various types of knowledge to improve KD. Methods in [34] argued that the soft label produced by **T**, *i.e.*, the classification probabilities, can provide richer information. Then, the distillation target is further extended to hidden layer features [35] and visual attention maps [36]. Except for distilling with model compression, knowledge distillation is also proved to be effective when the teacher and the student have identical architectures, i.e., self-distillation [37, 38], which transfers the knowledge between the same model structures. Knowledge distillation has also been applied in other areas such as semisupervised learning [15], curriculum learning [39], and neural style transfer [40].

RETRACTED

## 3. Incompatibility between Network Representation and Classification

As described above, network representation learning is “incompatible” with classifier learning in long-tailed classification that it is hard to achieve good results by learning jointly. In this section, we conduct ablations to further illustrate this problem. To clarify, in the following paper, instance-balanced sampling refers to sampling strategy that each training image has an equal probability to be selected and class-balanced sampling [9, 19] refers to images of each class, which has an equal probability to be selected.

A recent work [12] shows to us that the classifier's weight norm for different classes obeys a similar distribution with the number of samples in each class when performing instance-balanced training.  Figure 1 exhibits the **L2** norm of classifier weights with class indexes sorted by a descending order with respect to the number of instances in each class. As illustrated in the figure, consistent with conclusions in [12], if a class has more samples than other classes, its corresponding weight norm in the classifier is also larger than others with high probability and vice versa (orange line). But when applying class-balanced training to the classifier in the decouple method [12], the weight norm's distribution of all classes becomes more likely to uniform distribution (green line). We try to apply balanced sampling during the whole training process and visualize its classifier's weight norm (blue line), finding that it is very close to that of the decouple method, which means learning jointly with class-balanced sampling can also optimize the classifier into a good status. Then here comes a question: *why not directly use a class-balanced training strategy for jointly learning representation and classifier?*

It seems that class-balanced sampling is an optimal strategy that can achieve better classifiers than instance-balanced sampling and improve the performance of training models on the long-tailed dataset. However, results show that class-balanced sampling only brings limited improvement (from 35.7 to 36.5), as shown in the left column of Table 1. We explain it as the inferior quality of representation for a class-balanced model and following experiments further verify our claim.

We first train two models with instance-balanced strategy and class-balanced strategy on ImageNet-LT, respectively. Then classifiers of the two models are reinitialized and retrained on a different dataset (Places-LT) with their backbone (representation) fixed. During the classifier retraining process, class-balanced sampling is used. As class-balanced sampling can learn an optimal classifier, if one model shows clearly performance gain than another, then its quality of representation should be better than another. As shown in Table 1, the instance-balanced backbone shows a higher accuracy than class-balanced backbone (25.2% vs 22.1%), which indicates that instance-balanced sampling achieves better representations than class-balanced sampling. The experiment further demonstrates the “incompatibility” between representation learning and classifier learning as we have discussed.

RETRACTED

## 4. Methods

For long-tailed recognition, the training dataset follows an imbalance distribution over classes. As for the lack of training samples in tail classes, the result model tends to exhibit underfitting on few-shot classes. Existing methods focus on improving representation learning or classifier learning to promote the model performance on long-tailed datasets, but improvements in one aspect usually affect the other's performance, which is defined as “incompatibility” problem. To overcome this problem, we introduce our *multiexperts distillation* and *channel activation-based distillation* in this section. Through our approach, representation absorbs knowledge for different classes from expert models; meanwhile, class-balanced sampling guarantees that with the learned feature, there will be a good classifier to correctly classify our input images.

### 4.1. Preliminary

The knowledge distillation (KD) method typically employs a student *S*(·) to learn from a well-trained teacher model *T*(·), aiming at reproducing the predictive capability of *T*. In other words, given an image-label pair (*x*, *y*), *T* will make a prediction ${\hat{y}}^{T}=T\left(x\right),$ and *S* is trained with the purpose of outputting similar result as ${\hat{y}}^{T}$. Here, the prediction made by *S* is denoted as ${\hat{y}}^{S}=S\left(x\right)$.

To achieve this goal, KD targets at exploring a way to extract the information contained in a CNN model and then push the information of *S* to be as close to that of *T* as possible. Accordingly, the loss function of KD can be formulated as

(1) $$\begin{array}{c} {ℒ}_{KD}=d\left(\psi \left(T\left(\cdot \right),\Theta_{T}\right),\psi \left(S\left(\cdot \right),\Theta_{S}\right)\right), \end{array}$$

where Θ_*T*_ and Θ_*S*_ are the trainable parameters of *T* and *S*, respectively. *ψ*(·, ·) is the function that helps define the knowledge of a particular model, and *d*(·, ·) is the metric to measure the distance between the knowledge of two models.

Note that only Θ_*S*_ in Equation (1) is updated, since *T* is assumed to have already been optimized with ground truth. Then, the student network is trained to minimize the combination of task loss and KD loss:

(2) $$\begin{array}{c} {ℒ}_{S}=\phi \left(y,{\hat{y}}^{S}\right)+\lambda {ℒ}_{KD}, \end{array}$$

where *ϕ*(·, ·) is a task loss function, *e.g.*, softmax cross-entropy loss in classification, bounding box regression loss in detection.  *λ* is a loss weight hyperparameter to balance these two terms.

RETRACTED

### 4.2. Multiexperts Distillation

Formulation. Formally, given a dataset *D* with *C* classes, we split the entire dataset into *L* subsets {*D*_1_, *D*_2_,…, *D*_*L*_} with {*C*_1_, *C*_2_,…, *C*_*L*_} classes in each of them. Specifically, *n*_*D*_*i*__^*j*^ denotes the number of training samples for class *j* in subset *D*_*i*_. Different from traditional KD methods that the teacher is a deeper, larger model than the student, our experts are exactly the same model with the student but with various performances on different subdatasets. The loss function of KD can be formulated as

(3) $$\begin{array}{c} {ℒ}_{S}=\phi \left(y,{\hat{y}}^{S}\right)+\overset{L}{\underset{i=1}{\sum }}\lambda_{i}d\left(\psi_{D_{i}}\left(T_{i}\left(\cdot \right),\Theta_{T_{i}}\right),\psi_{D_{i}}\left(S\left(\cdot \right),\Theta_{S}\right)\right), \end{array}$$

where *ψ*_*D*_*i*__(·, ·) indicates the knowledge that is only calculated with training samples in subset *D*_*i*_.

Note that class-balanced sampling is used as the sampling strategy when training student model with knowledge distillation process. As discussed in Section 3, jointly learning with class-balanced sampling strategy can optimize the classifier into a good status. The combination of these two terms (KD and class-balanced sampling) makes the final model perform better on both representation and classifier, resulting in higher accuracy on long-tailed scenarios.

In this work, we treat feature maps of a CNN model as the underlying knowledge. Generally, a model can be divided into a set of *K* blocks, and the output of each block is considered as a hidden feature map. For an input batch, the K feature maps of a network can be denoted as {*f*_*k*_ ∈ *R*^*b*×*c*×*h*×*w*^}_*i*=1_^*K*^, where *b* is the batch size, *c* is the number of channels, and *h* and *w* are the height and width of the feature spatial dimension, respectively. For *d*(·, ·), we use *l*_2_ distance: *d*(*a*, *b*)=||*a* − *b*||_2_^2^ to measure the difference between feature representations. Accordingly, to transfer representation knowledge from *L* experts to one student, Equation (3) can be simplified as

(4) $$\begin{array}{c} L_{S}=\phi \left(y,{\hat{y}}^{S}\right)+\overset{L}{\underset{i=1}{\sum }}\overset{K}{\underset{k=1}{\sum }}\lambda_{i}{\left|\left|\psi_{D_{i}}\left(f_{k}^{T_{i}}\right)-\psi_{D_{i}}\left(f_{k}^{S_{i}}\right)\right|\right|}_{2}^{2}. \end{array}$$

An overview of the framework is presented in Figure 2.

RETRACTED

Design of expert. In multiexperts knowledge distillation, one important thing is how to find *L* experts to supervise the student model. For a long-tailed problem, we specially design experts according to number of training samples in each category. Specifically, the long-tailed dataset *D* with *C* classes will be divided according to threshold values: {*γ*_1_, *γ*_2_,…, *γ*_*L*−1_}. After splitting, each subset *D*_*i*_ satisfies *γ*_*i*−1_ ≤ *n*_*D*_*i*__^*j*^ < *γ*_*i*_, where *n*_*D*_*i*__^*j*^ denotes training samples for class *j* in *D*_*i*_. Then, *L* experts {*T*_1_, *T*_2_,…, *T*_*L*_} will be trained and each expert should be well performed on one of *D*_*i*_. Experts can be trained with other state-of-the-art long-tailed methods using the whole dataset or trained from the scratch with only subset samples. For a specific subset *D*_*i*_, we will find a model that performs well on *D*_*i*_ as an expert model *T*_*i*_. Notice that we do not guarantee an expert performs well on the whole dataset, but it should be skilled at one of the subsets. This is motivated by the problem that existing methods always sacrifice the accuracy of some dominant classes to improve the accuracy of tail classes. These *L* experts contain better representations on the *L*  subsets *D*_*i*_ and knowledge distillation is used to integrate all of the representation knowledge to one student model.

### 4.3. Channel Activation-Based Distillation

Once we use knowledge distillation to transfer long-tailed representations from experts to students, using *L*_2_ distance to measure differences between feature maps is a direct but naive way. Considering the representation map of a well-trained model, there may be channels, which contain less information or even contain noise information. If we could find out channels that obtain most useful information for distillation, the learning effectiveness should be improved. As a result, a novel channel activation-based KD is therefore proposed to enhance multiexperts knowledge distillation.

Our approach is motivated by an interesting observation that, in a well-trained network, for its feature maps *f*_*k*_, the activation intensity of channels performs differently. To better illustrate, we take out representations of the final block in ResNet-20, following with an average pool to obtain a vector with 64 values. Thus, each value of the vector reflects the activation intensity of a channel. Each representation is an average feature map among one category over CIFAR-100 training set.  Figure 3 shows the representation vectors and each banner refers to features averaged in different categories. We can see that some pixels have a brighter color, representing that the corresponding channel is highly activated, while others are not. Furthermore, the distribution of activation intensity performs differently among different classes. Based on the observation, we regard that channels with higher activation intensity contain more important knowledge and those with lower activation intensity have less knowledge or even noise information. Therefore, to improve the knowledge transfer performance, we should put more attention on the highly activated knowledge.

RETRACTED

Define *σ*_*c*_(·, *α*) as the function to extract channels with the highest activation intensity in class *c*. *α* is the hyperparameter to control how many channels are selected, *e.g.*, *α*=0.9 means that 90% channels are used in knowledge distillation and activation of these selected channels is higher than abandoned ones. *σ*_*c*_(·, *α*) is achieved by a statistically analyzed well-trained student model in advance. Activation maps will be averaged among all samples on class *c* and channel indexes will be sorted and recorded in terms of activation intensity value in a descending order. *σ*_*c*_(·, *α*) selected channels through recorded indexes and hyperparameter *α*. With the help of *σ*_*c*_(·, *α*), Equation (4) can be rewritten as

(5) $$\begin{array}{c} \underset{\Theta_{S}}{\min}L_{S}=\phi \left(y,{\hat{y}}^{S}\right)+\lambda \overset{l}{\underset{i=1}{\sum }}\overset{C_{i}}{\underset{c=1}{\sum }}\overset{k}{\underset{k=1}{\sum }}{\left\|\psi_{D_{i}}\left(\sigma_{c}\left(f_{k}^{T_{i}},\alpha \right)\right)-\psi_{D_{i}}\left(\sigma_{c}\left(f_{k}^{S_{i}},\alpha \right)\right)\right\|}_{2}^{2}. \end{array}$$

With the channel activation-based KD approach, the student model is capable of distilling knowledge from experts effectively and efficiently and achieves representations that perform good for both head classes and tail classes.

## 5. Experiments

### 5.1. Experimental Settings

  Dataset: we evaluate our proposed method on three large-scale long-tailed datasets, including ImageNet-LT [10], Places-LT [10], and iNaturalist-2018 [21]. ImageNet-LT and Places-LT are long-tailed versions of the original dataset: ImageNet-2012 [2] and Places-2 [25], by artificially sampling from them. Overall, ImageNet-LT contains 115.8 K images from 1000 categories, with the number of images in each class range from 1280 to 5. Places-LT has 184.5 K images from 365 categories, with the maximum of 4980 images per class and minimum of 5 images per class. iNaturalist-2018 classification datasets are large-scale real-world datasets that suffer from the extremely imbalanced label distribution with 437.5 K images from 8,142 categories.
  Evaluation metrics: to better examine the performance, following [10], except for reporting accuracy on whole dataset, we evaluate results according to three sets of classes: *Many-shot* (more than 100 images), *Medium-shot* (20 to 100 images), and *Few-shot* (less than 20 images). We follow the settings in [10–12] for our method on different datasets.
  Implementation details: PyTorch framework is used for all experiments. For ImageNet-LT, we employ a scratch ResNet-10 as our backbone network. On Places-LT, to make a fair comparison with results in [10], ResNet-152 is used and it is well pretrained on ImageNet. ResNet-50 is used for iNaturalist-2018 following settings in [12]. As for all experiments, if not specified, an SGD optimizer with momentum 0.9, batch size 512, weight decay 0.0005, and cosine learning rate schedule gradually decaying from 0.2 to 0 is used. The image resolution is 224 × 224 and the network is trained for 90 epochs. The distillation loss is calculated with the output feature maps before average pool and *α* is set to 0.9. Corresponding to evaluate with three sets of classes (many shot, medium shot, and few shot), the training dataset *D* is also split into three parts following the same protocol as evaluation set, and three experts {*T*_1_, *T*_2_, *T*_3_}, responsible for each part of the new set, are used as teachers in the knowledge distillation process. {*λ*_1_, *λ*_2_, *λ*_3_} is set to be 1*e*^−3^, 1*e*^−4^, 1*e*^−4^, respectively, and the principal to choose *λ*_*i*_ is to balance all the loss terms into the same order of magnitude.

RETRACTED

### 5.2. Ablation Studies

In this section, we conduct ablations to show the effectiveness of the proposed method. A well-trained model on many-shot subsets (many-shot model) and a model trained with OLTR [10] are used as our experts in all sections.

#### 5.2.1. Ablation on Different Experts

In this section, we show the influence of using different expert models. According to our design, for the three subsets, many-shot, medium-shot, and few-shot, three experts are needed and with each expert, there are three choices: *plain model* (model trained from scratch with whole dataset), *subset model* (model trained from scratch with certain subset data), and *OLTR model* (any long-tailed methods can be used, and we take OLTR as an example).

Experiments of using different experts are shown in Table 2. Except for our common settings used in other sections, which uses experts with best performance for each subset (many-shot model for many-shot and OLTR for medium-shot, few-shot), we also apply our approach with three subset models as experts, which are experts with lowest accuracy among all the choices. Furthermore, since there are totally 27 possible expert combinations choices, which are too many to show, we exhibit an average result over 5 randomly chosen combinations. The random combinations are choices of designed experts with accuracy between our common settings and settings with three subset models. The results consistently show that when applying the distillation approach, using designed experts with better performance will result in higher accuracy.

Furthermore, as our experts are designed to supervise subsets, which are divided according to class sample numbers to fit into the long-tail problem, there are also more direct and simple ways that just randomly split the dataset and use each subset to train an expert. We also compare our approach with this *randomly splitting strategy*. Unlike our design, in random strategy, the whole dataset is split into three pieces taking no account of how many samples in each category. Each subset is used to train an expert and three experts are used to supervise a student. The process is repeated 5 times and an average result is shown in the last line of Table 2. The randomly splitting strategy achieves a worse performance than our approach, which indicates the preponderance of our design.

#### 5.2.2. Instance-Balanced Sampling vs Class-Balanced Sampling

As described in Sections 3 and 4, the proposed method learns knowledge from experts to improve network representation learning; meanwhile, class-balanced sampling is applied together with it to take care of classifier learning. The combination of these two parts ensures that representation and classifier can be jointly learned. In order to show the strength of using class-balanced strategy, we conduct ablations in Table 3 by exhibiting comparison results of applying class-balanced sampling and instance-balanced sampling with our approach on ImageNet-LT. From the results, class-balanced strategy always comes up with higher performance on medium-shot, few-shot, and overall accuracy.

Furthermore, we also conduct experiments to demonstrate that knowledge distillation can improve the representation learning quality. Similar to experiments in Section 3, we retrain the classifier of ImageNet-LT results on another dataset: Places-LT and the performance on Places-LT can reflect the representation quality of different strategies. As shown in Table 4, our approach achieves a higher accuracy after fine-tuning the classifier on Places-LT, which illustrates that with the help of knowledge distillation, a model can learn better representations.

RETRACTED

#### 5.2.3. Ablation on Knowledge Distillation Settings

As the proposed method consists of various components: multiexperts knowledge distillation and channel activation-based learning strategy. In this section, we investigate ablations on the contribution of each part and show the results in Table 5. The three rows in this table refer to applying with traditional one teacher knowledge distillation, applying with multiexperts knowledge distillation, and applying with channel activation-based knowledge distillation, respectively.

The first column is the plain ResNet-10 model that directly trained on ImageNet-LT. Compared with simply applying knowledge distillation with one expert model (OLTR model), the proposed multiexperts approach increases from 37.1% to 38.6%. Furthermore, combined with channel activation-based strategy, there is still an improvement of 0.6% in accuracy (38.6% to 39.2%).

### 5.3. Comparison with State-of-the-Art Methods

In this section, we compare the performance of our approach with other recent state-of-the-art methods on three common long-tailed benchmarks: ImageNet-LT, Places-LT, and iNaturalist. Similar to settings in ablations, for all the experiments of our approach, we use a many-shot model to supervise a many-shot subset; meanwhile, ours with decouple means Decouple (cRT) is used as an expert for medium-shot as well as few-shot subsets and ours with OLTR means OLTR is used for supervising medium-shot and few-shot. All the results for other work are copied from their paper or reproduced with author's code.

ImagetNet-LT: Table 6 represents the classification results for ImageNet-LT. For the state-of-the-art Decouple methods, we reproduce the results according to the author's codebase and two training settings are used, which corresponds to cRT and *τ*-normalized classifier learning strategy. Results show that our proposed method achieved the highest performance (43.9%) on overall accuracy.

Places-LT: for experiments on Places-LT, we follow the settings in [10] starting from a pretrained ResNet-152 on ImageNet [2] and fine-tune the backbone model with instance-balance sampling as a plain model. Results are shown in Table 7 that the our method outperforms other state-of-the-art approaches, including Lifted Loss [41], Focal Loss [13], Range Loss [14], FsLwf [42], OLTR [10], BALMS [43], and Decouple [12]. For overall accuracy, our method improves the plain model with 8.5% in accuracy.

iNaturelist. We further evaluate the proposed method on the iNaturalist dataset. From Table 8, the experimental results show consistency with ImageNet-LT and Places-LT cases. Our proposed method surpasses OLTR and Decouple (*τ*-normalized) method with 3.4% and 1.6% in overall accuracy, respectively. Furthermore, the accuracy of medium-shot and few-shot classes also performs the best among other competitors.

RETRACTED

### 5.4. Confusion Matrix Analysis

In this section, we provide the confusion matrix analysis on the three commonly used long-tailed datasets: ImageNet-LT, Places-LT, and iNaturalist. We compare the recall and precision calculated by the confusion matrix with the state-of-the-art long-tailed approach Decouple [12] and show the results in Table 9. As shown in the table, for precision and recall metric, our approach consistently shows its superiority on the long-tailed dataset compared with the state-of-the-art method.

## 6. Conclusion

In this paper, we discuss the incompatibility between network representation learning and classifier learning when training deep neural networks on a long-tailed scenario. A multiexperts knowledge distillation method is therefore proposed to jointly learn representation and classifier simultaneously. Furthermore, to further improve the performance, a channel activation-based learning strategy is also proposed. Evaluation results and ablation studies on three long-tailed benchmarks indicate the efficiency and effectiveness of the proposed method.

## Figures and Tables

**Figure 1:** Classifier weight norm for ResNet-10 trained on ImageNet-LT. The class indexes are sorted by descending values of class sample numbers.

**Figure 2:** Framework overview of the proposed method. Here, training datasets are split into three subsets and three experts are used as teachers. Each expert is responsible for transferring knowledge from its corresponding subset into a student model. The knowledge is transferred between feature maps and only channels with high activation intensity, which we consider as containing more knowledge, will be used for distillation. Details about filtering channels are introduced in Section 4.3.

**Figure 3:** Visualization of features where each one is a vector averaged among one category on CIFAR-100. Each banner is taken from three different classes. Brighter color corresponds to a higher activation intensity.

**Table 1:** Comparison feature quality between class-balanced sampling (CBS) and instance-balanced sampling (IBS). ResNet-10 models are trained on ImageNet-LT (I-LT), and then classifiers are retrained with class-balanced sampling on Places-LT (P-LT).

Representation		Classifier	
Strategy	ImageNet-LT	Strategy	Places-LT
IBS	35.7	CBS	25.2
CBS	36.5	CBS	22.1

**Table 2:** Ablation of using different experts while applying the proposed method.

Model	Many-shot	Medium-shot	Few-shot	Acc
ResNet-10	>100	≤100 and >20	≤20	
Plain model	56.8	25.7	3.6	34.6
Many-shot model	57.9	—	—	—
Medium-shot model	—	32.5	—	—
Low-shot model	—	—	10.6	—
OLTR [10]	43.2	35.1	18.5	35.6
Ours with many-shot/OLTR/OLTR	54.0	34.1	17.4	39.2
Ours with many-shot/medium-shot/low-shot	54.4	28.7	8.9	36.9
Average over combination of designed experts	53.7	32.9	14.5	37.2
Average over randomly splitting strategy	48.3	27.6	8.7	36.4

Ours with A/B/C refers to A, B, and C which are used as expert models to supervise many-shot/medium-shot/few-shot subsets, respectively. Experiments are performed on ImageNet-LT with ResNet-10.

RETRACTED

**Table 3:** Ablation of our approach using instance-balanced sampling (IBS) and class-balanced sampling (CBS) with ResNet-10 on ImageNet-LT.

Shot	IBS	CBS
Many-shot model	**54.9**	54.0
Medium-shot model	32.9	**34.1**
Few-shot model	16.8	**17.4**
Overall	37.5	**39.2**

Bold values are the highest results in each line.

**Table 4:** Ablation of representation quality with our method. ResNet-10 is first trained on ImageNet-LT (I-LT). Classifiers are retrained on Places-LT (P-LT).

Representation		Classifier	
Strategy	ImageNet-LT	Strategy	Places-LT
IBS	35.7	CBS	25.2
CBS	36.5	CBS	22.1
Ours with IBS	37.5	CBS	28.2
Ours with CBS	39.2	CBS	27.8

**Table 5:** Ablation of knowledge distillation settings on ImageNet-LT.

Distillation	—	√	√	√	√
Multiexperts	—	—	√	—	√
Channel activation	—	—	—	√	√
Acc	35.7	37.1	38.6	37.8	**39.2**

**Table 6:** Long-tailed classification results on ImageNet LT.

Model	Many-shot	Medium-shot	Few-shot	Acc
ResNet-10	>100	≤100 and >20	≤20	
Plain model	56.8	25.7	3.6	34.6
Many-shot model	**57.9**	—	—	—
Lifted loss^†^ [41]	35.8	30.4	17.9	30.8
Focal loss^†^ [13]	36.4	29.9	16	30.5
Range loss^†^ [14]	35.8	30.3	17.6	30.7
FsLwf^†^ [42]	40.9	22.1	15	28.4
OLTR^*∗*^ [10]	43.2	35.1	18.5	35.6
BALMS^†^ [43]	50.3	39.5	25.3	41.8
Decouple (cRT)^*∗*^ [12]	52.3	39.5	23.2	42.1
Decouple (*τ*-normalized)^*∗*^ [12]	51.9	38.3	22.5	40.6
Ours with OLTR	54.0	34.1	17.4	39.2
Ours with decouple	54.9	**39.6**	**23.4**	**43.9**

^†^Results directly copied from Ref. [10]. ^*∗*^Results reproduced with author's code.

**Table 7:** Long-tailed classification results on Places-LT, starting from an ImageNet pretrained ResNet-152.

Model	Many-shot	Medium-shot	Few-shot	Acc
ResNet-152	>100	≤100 and >20	≤20	
Plain model	45.5	27.8	8.5	30.2
Many-shot model	46.4	—	—	—
Lifted loss^†^ [41]	41.1	34.8	22.4	34.6
Focal loss^†^ [13]	41.1	35.4	24	35.2
Range loss^†^ [14]	41.1	35.4	23.2	35.1
FsLwf^†^ [42]	43.9	29.9	29.5	34.9
OLTR^*∗*^ [10]	42.2	38.1	17.8	35.3
BALMS^†^ [43]	41.2	39.8	31.6	38.7
Decouple (cRT)^*∗*^ [12]	41.6	39.4	29.2	38.1
Decouple (*τ*-normalized)^*∗*^ [12]	37.8	40.7	31.8	37.9
Ours with OLTR	43.8	37.8	17.5	37.5
Ours with decouple	41.5	40.9	32.2	38.7

^†^Results directly copied from Ref. [10]. ^*∗*^Results reproduced with author's code.

RETRACTED

**Table 8:** Long-tailed classification results on iNaturalist-2018.

Model	Many-shot	Medium-shot	Few-shot	Acc
ResNet-50	>100	≤100 and >20	<20	
Plain model	73.5	65.2	59.5	63.6
Many-shot model	74.6	—	—	—
OLTR^*∗*^ [10]	65.9	66.3	63.6	65.4
Decouple (cRT)^*∗*^ [12]	66.2	67.3	66.8	67.0
Decouple (*τ*-normalized)^*∗*^ [12]	65.4	66.8	66.9	67.2
Ours with OLTR	68.7	66.2	63.5	67.4
Ours with decouple	69.4	69.3	67.6	68.8

**Table 9:** Precision and Recall analysis on long-tailed dataset.

Dataset	Precision-decouple [12]	Precision-ours	Recall-decouple [12]	Recall-ours
ImageNet-LT	69.9	72.8	62.0	66.9
Places-LT	58.6	62.6	53.5	58.7
iNaturalist	73.9	75.1	71.7	74.8

## Data Availability

All the data used in this paper are publicly available.
